RETRACTED

# Expression and Clinical Trends of Pct Combined with Lactate Clearance in Sepsis

**DOI:** 10.1155/2022/4382671

**Published:** 2022-05-30

**Authors:** Shigang Li, Zhe Chen, Weifeng Yan

**Affiliations:** Beijing Haidian Hospital, Beijing 100080, China

## Abstract

**Objective:**

To study the expression and clinical trend of procalcitonin (Pct) + lactate clearance in sepsis.

**Methods:**

A total of 63 septic shock patients enrolled in our hospital from March 2018 to March 2021 were recruited as group A, and the 87 septic patients admitted during the same period were recruited as group B. The Pct, lactic acid, and lactate clearance were compared between the two groups.

**Results:**

The Pct and lactic acid in group A were higher than those in group B at the time of diagnosis, 1 d, 2 d, and 3 d after treatment, but the lactate clearance rate at 1 d, 2 d, and 3 d after treatment was lower than that in group B (*P* < 0.05). The Pct and lactate at the time of diagnosis, 1 d, 2 d, and 3 d after treatment in the good prognosis group were lower than those in the poor prognosis group, but the lactate clearance rate at 1 d, 2 d, and 3 d after treatment was higher than that in the poor prognosis group (*P* < 0.05). Disease severity and prognosis were positively correlated with Pct and lactate, but negatively correlated with lactate clearance rate (*P* < 0.05).

**Conclusions:**

Pct and lactate clearance rate might serve as accurate predictors of the severity of sepsis and prognosis. It merits promotion in clinical setting.

## 1. Introduction

Sepsis, as a common clinical systemic inflammatory response syndrome, is one of the acute and critical illnesses. It is often triggered by the damaged circulatory system caused by infections, resulting in hypoperfusion of tissues and multiple organ failure. Septic shock is a common and severe type of sepsis that complicates with circulatory and cell metabolism disorders. Delayed detection and treatment might lead to life-threatening conditions [1, 2]. Statistics show that the septic shock-related death is up to 30–70% [3]. Hence, it is of great significance to seek an effective means to assess the severity and prognosis of the disease. Despite the wide use of the sequential organ failure assessment (SOFA) in clinical evaluation, its application is restricted due to multiple scoring items, time-consuming properties, and susceptibility to subjective factors. A cascade of evidence has confirmed that inflammatory markers such as procalcitonin (Pct), lactate, and lactate clearance rate are linked to the disease, and their levels reflect the patient's tissue perfusion and infection, yet its underlying mechanism is poorly understood by now [4, 5]. According to the Chinese Sepsis Guidelines in 2014, sepsis is categorized into sepsis, severe sepsis, and septic shock according to the severity of the disease [6]. The guidelines recommend the use of Pct, C-reactive protein, IL-6, and other inflammatory factors as markers of disease progression in patients with sepsis. Blood lactate is a product of glucose metabolism, and its subsequent metabolism is highly dependent on oxygen. If the tissue perfusion is low and oxygen supply is insufficient, its metabolic efficiency will be seriously affected [7]. In patients with sepsis, due to the systemic inflammatory response, the direct response indicators of the severity of the disease are closely related to the level of tissue perfusion and oxygen supply [8]. Armed with this knowledge, blood lactate, and Pct were used as markers for the evaluation of the condition and prognosis of patients with sepsis in the present study, and their feasibility was analyzed from the trend. Herein, this study was conducted to investigate the expression and clinical trends of Pct combined with lactate clearance in sepsis.

RETRACTED

## 2. Materials and Methods

### 2.1. Baseline Data

A total of 63 septic shock patients enrolled in our hospital from March 2018 to March 2021 were selected as group A, and the 87 septic patients admitted during the same period were recruited as group B. Group A had 33 males and 30 females, aged 36–74 years, with an average age of (51.26 ± 3.28) years; group B had 46 males and 41 females, aged 34–72 years, with an average age of (51.77 ± 3.51) years. The baseline data in the two groups were well balanced.

### 2.2. Inclusion and Exclusion Criteria

#### 2.2.1. Inclusion Criteria

Inclusion criteria were as follows: (1) patients who met the diagnosis criteria in the Chinese Guidelines for Emergency Treatment of Sepsis/Septic Shock [6]; patients who presented with fever or hypothermia, increased heart rate, shortness of breath, poor mental status, hyperglycemia, inflammatory markers, hemodynamic changes, organ failure, hypotension or (and) lactate clearance ≥1 mmol/L or (and) adequate fluid resuscitation, urine output remains <0.5 ml/(kg·h) for at least 2 hours, or (and) acute lung injury not caused by pneumonia and PaO_2_/FiO_2_ < 250 mmHg, or (and) acute lung injury due to pneumonia and PaO_2_/FiO_2_ < 200 mmHg, or (and) serum creatinine level >176.8 *μ*mol/L, or (and) bilirubin >34.2 *μ*mol/L, or (and)) platelet count <100 × 10^9^/L or (and) coagulation disorder, etc. and confirmed by examinations; (2) patients who signed informed consent, and the study was approved by the Ethics Committee of Beijing Haidian Hospital, No.HD7703; and (3) patients who had complete medical records and did not withdraw from the trial midway.

RETRACTED

#### 2.2.2. Exclusion Criteria

Exclusion criteria were as follows: (1) patients with neurological diseases, malignant tumors, hematological diseases, and urinary system diseases; (2) the survival was less than 2 weeks; and (3) nervous system diseases, etc., that affected the assessment of prognosis.

### 2.3. Methods

The cubital venous blood (4 ml) was drawn in the morning, centrifuged at 4000 r/min for 10 min, isolated, and stored at −20°C for testing. A chemiluminescence analyzer (German Brahms company, LuamtLB-9507) and supporting reagents were used to measure Pct in strict accordance with the instructions; a blood gas analyzer (Siemens RAPIDPoint 500) was used to measure lactate strictly in accordance with the enzyme electrode method; lactate clearance rate = (lactate at diagnosis−lactate after treatment)/lactate at diagnosis *∗* 100.00%.

After diagnosis, both groups received targeted anti-infection, fluid resuscitation, anticoagulation, mechanical ventilation, vasoactive drugs, renal replacement, and other treatments.

### 2.4. Support Treatment

The Chinese medicine Fusu Decoction (provided by Beijing Haidian Hospital preparation room, 0.4 g/capsule) was given for support treatment, 4 capsules each time, orally or by nasal feeding after dissolving in cold water, 3 times a day; the drug composition is American ginseng, astragalus, raw rhubarb, gypsum, *Ophiopogon japonicus*, salvia, red peony, etc.

### 2.5. Outcomes

1. The Pct and lactate at diagnosis, 1 d, 2 d, and 3 d after treatment, and the lactate clearance rate at 1 d, 2 d, and 3 d after treatment in groups A and B were compared.
2. 150 patients were followed up, of whom 133 survivors were classified as the good prognosis group, and the other 17 deceased patients were classified as the poor prognosis group. Lactic acid and lactate clearance at 1 d, 2 d, and 3 d after treatment were compared.
3. Pearson analysis was performed to analyze the correlation between Pct, lactate, lactate clearance rate, and disease severity and prognosis.

### 2.6. Statistical Analysis

Data were expressed as the mean ± standard deviation and cases (%). Statistical analysis was performed using SPSS 22.0 (IBM, Armonk, NY, USA). Differences between groups were compared using Student's *t*-test and chi-square tests, and Pearson analysis was performed to analyze the correlation. A *P* value < 0.05 was considered statistically significant.

## 3. Results

### 3.1. The Pct, Lactate, and Lactate Clearance Rates of the Two Groups at Different Times

The Pct and lactic acid in group A were higher than those in group B at the time of diagnosis, 1 d, 2 d, and 3 d after treatment, but the lactate clearance rate at 1 d, 2 d, and 3 d after treatment was lower than that in group B (*P* < 0.05) (see Table 1).

RETRACTED

### 3.2. The Pct, Lactate, and Lactate Clearance in Patients with Different Prognosis

The Pct and lactate at the time of diagnosis, 1 d, 2 d, and 3 d after treatment in the good prognosis group were lower than those in the poor prognosis group, but the lactate clearance rate at 1 d, 2 d, and 3 d after treatment was higher than that in the poor prognosis group (*P* < 0.05) (see Table 2).

### 3.3. Correlation of Pct, Lactate, and Lactate Clearance Rate with Disease Severity and Prognosis

Disease severity and prognosis were positively correlated with Pct and lactate, but negatively correlated with lactate clearance rate (*P* < 0.05) (see Table 3).

## 4. Discussion

Recent years witnessed a stubbornly high prevalence and fatality rate of sepsis worldwide, with the global figure exceeding 19 million per year, and the death toll of 5.3 million [7]. If timely diagnosis and treatment were not provided, the disease would progress even to shock that is a life-threatening condition. Therefore, clinical endeavors are urgent to enhance diagnosis and treatment of diseases by seeking more convenient, faster, and more accurate indicators [8, 9].

Pct, an immunoregulatory protein, is a common indicator for severe infection and is of tremendous significance in evaluating the outcome of infection; lactate, as a compound, plays a role in various physiological mechanisms and is strongly related to inflammatory responses [10]. However, there are few reports on the correlation between Pct and lactate clearance rate and diseases. This study showed that the Pct and lactic acid in group A were higher than those in group B at the time of diagnosis, 1 d, 2 d, and 3 d after treatment, but the lactate clearance rate at 1 d, 2 d, and 3 d after treatment was lower than that in group B. The Pct and lactate at the time of diagnosis, 1 d, 2 d, and 3 d after treatment in the good prognosis group were lower than those in the poor prognosis group, but the lactate clearance rate at 1 d, 2 d, and 3 d after treatment was higher than that in the poor prognosis group. Disease severity and prognosis were positively correlated with Pct and lactate but negatively correlated with lactate clearance rate. All these suggest that with the aggravation of the disease, the Pct level of patients increases, and the lactate clearance rate decreases. In addition, compared with the dead patients, the Pct of the survivors is lower and the lactate clearance rate is higher, suggesting that the Pct and lactate clearance rate might be a key indicator for evaluating disease severity and prognosis. Due to hypoxia and tissue hypoperfusion in patients with sepsis, the anaerobic glycolysis of glucose increases and the production of lactic acid increases significantly. When lactic acid exceeds 2 mmol/L, it goes beyond the liver's clearance capacity, which can cause lactic acid accumulation and hyperlactatemia that are important indicators of hypoxia and shock; when it exceeds 4 mmo/L, the mortality rate of patients with sepsis is significantly increased [10, 11]. Therefore, dynamic monitoring of blood lactate level and calculation of lactate clearance rate are of great significance for evaluating the severity of the disease and judging the prognosis.

RETRACTED

As previously noted, lactic acid is a product of glucose metabolism, and the lactic acid secreted by glucose metabolism can be decomposed into other substances in sufficient oxygen supply conditions, so the lactic acid level is relatively low under normal circumstances [11–13]. Once acute and critical illness-related hypoxia occurs, pyruvate after glucose metabolism could hardly complete the metabolic process due to hypoxia. Lactic acid accordingly accumulates in the body and increases the risk of lactic acidosis, and the lactate clearance rate indicates the oxygen supply and consumption of the body [14–16]. Pct, a precursor of calcitonin, is composed of multiple amino acids and tends to increase once exposed to bacterial infection and is correlated with the severity of the disease. Hence its expression reflects the infection status [17, 18]. Moreover, the traditional Chinese medicine compound preparation for the treatment of sepsis-Fusu decoction in the present study is mainly composed of American ginseng, *Astragalus*, *Ophiopogon japonicus*, Scrophulariaceae, gypsum, Anemarrhena, licorice, *Coptis chinensis*, buffalo horn, *Salvia miltiorrhiza*, red peony root, *rehmannia glutinosa*, forsythia, pale bamboo leaves, and rhubarb. The combination of various medicines can clear the unhealthy qi and restore yin and yang dynamic balance.

## 5. Conclusion

Pct and lactate clearance rate can accurately predict the severity of sepsis and evaluate the prognosis. It merits promotion in clinical setting.

## Figures and Tables

**Table 1:** The Pct, lactate, and lactate clearance rates of the two groups at different times.

Groups	Pct (ng/ml)				Lactate (mmol/L)				Lactate clearance rates (%)		
	At diagnosis	1 d after treatment	2 d after treatment	3 d after treatment	At diagnosis	1 d after treatment	2 d after treatment	3 d after treatment	1 d after treatment	2 d after treatment	3 d after treatment
Group A (*n* = 63)	3.12 ± 1.03	3.47 ± 1.14	3.88 ± 1.23	4.10 ± 1.35	3.74 ± 1.23	3.40 ± 1.13	3.26 ± 1.07	3.20 ± 1.05	6.35 ± 2.10	8.87 ± 2.94	10.24 ± 3.40
Group B (*n* = 87)	2.62 ± 0.86	2.77 ± 0.92	2.85 ± 0.94	3.11 ± 1.02	2.23 ± 0.74	1.95 ± 0.64	1.87 ± 0.61	1.81 ± 0.59	9.14 ± 3.03	10.52 ± 3.46	15.89 ± 5.26
*t*	3.233	4.157	5.813	5.116	9.355	9.970	10.073	10.310	6.293	3.067	7.467
*P*	0.002	0.001	0.001	0.001	0.001	0.001	0.001	0.001	0.001	0.003	0.001

RETRACTED

**Table 2:** Pct, lactate, and lactate clearance in patients with different prognosis.

Groups	Pct (ng/ml)				Lactate (mmol/L)				Lactate clearance (%)		
	At diagnosis	1 d after treatment	2 d after treatment	3 d after treatment	At diagnosis	1 d after treatment	2 d after treatment	3 d after treatment	1 d after treatment	2 d after treatment	3 d after treatment
Good prognosis group (*n* = 133)	2.38 ± 0.78	2.17 ± 0.70	2.03 ± 0.66	1.94 ± 0.62	3.06 ± 1.01	3.02 ± 0.96	2.95 ± 0.93	2.80 ± 0.91	7.03 ± 2.30	9.58 ± 3.13	10.97 ± 3.64
Poor prognosis group (*n* = 17)	3.95 ± 1.30	9.69 ± 3.22	3.55 ± 1.13	4.07 ± 1.33	3.65 ± 1.20	3.70 ± 1.22	3.84 ± 1.27	3.72 ± 1.22	−1.35 ± 0.44	−3.52 ± 1.16	−4.06 ± 1.35
*t*	7.157	23.391	8.133	11.316	2.219	2.663	3.553	3.766	14.945	7.894	7.740
*P*	0.001	0.001	0.001	0.001	0.028	0.009	0.001	0.001	0.001	0.001	0.001

**Table 3:** Correlation between Pct, lactate, lactate clearance rate, and disease severity and prognosis.

	Disease severity		Prognosis	
	*r*	*P*	*r*	*P*
Pct	0.698	0.005	0.763	0.002
Lactate	0.724	0.011	0.801	0.014
Lactate clearance rate	−0.559	0.003	−0.725	0.010

## Data Availability

The datasets used during the present study are available from the corresponding author upon reasonable request.
